# The Effect of Microwave Ablation Combined with Anti-PD-1 Monoclonal Antibody on T Cell Subsets and Long-Term Prognosis in Patients Suffering from Non-Small-Cell Lung Cancer

This article has been retracted.

**DOI:** 10.1155/2022/7095423

**Published:** 2022-09-26

**Authors:** Wenbo Yu, Jiewei Sun, Tao Wang, Yanan Du

**Affiliations:** ^1^Department of Respiratory and Critical Care Medicine, Yantai Yuhuangding Hospital, Yantai, Shandong 264001, China; ^2^Department of Interventional Therapy, Yantai Yuhuangding Hospital, Yantai, Shandong 264001, China; ^3^Department of Nuclear Medicine, Yantai Yuhuangding Hospital, Yantai, Shandong 264001, China

## Abstract

**Objective:**

This research is aimed at studying the effect of microwave ablation combined with the antiprogrammed death- (PD-) 1 monoclonal antibody on T cell subsets and long-term prognosis in patients suffering from non-small-cell lung cancer (NSCLC).

**Methods:**

Employing the random number table technique, a total of 122 NSCLC patients who received treatment at our hospital between May 2015 and June 2019 were selected and assigned to the observation group and the control group, and each group comprised 61 patients (*n* = 61). While the control group received only anti-PD-1 monoclonal antibody treatment, the observation group received microwave ablation in combination with anti-PD-1 monoclonal antibody. The clinical efficacy was observed for both groups. The levels of T cell subsets (CD3+, CD4+, and CD8+), serum tumor markers (squamous cell carcinoma antigen (SCCA), cytokeratin Ig fragment (CYFRA21-1), and serum carcinoembryonic antigen (CEA)), nuclear factor kappa B (NF-*κ*B), protease C (PKC), and mitogen-activated protein kinase (MAPK) mRNA expression between the two groups were compared. The frequency of adverse reactions was observed in both groups. The survival time of both the groups was recorded over the course of three years of follow-up. The Kaplan-Meier method was employed for analyzing the survival of both the control and the observation group.

**Results:**

The response rate (RR) of the observation group (80.33%) was considerably greater in comparison to that of the control group (62.30%) (*P* < 0.05). Following treatment, the observation group's levels of CD3+, CD4+, CD8+, SCCA, CyFRA21-1, and CEA and the mRNA expressions of NF-*κ*B, PKC, and MAPK were superior to those of the control group, with statistical significances (all *P* < 0.05). Between the two groups, there was no significant difference in the occurrence of adverse reactions (*P* > 0.05). The observation group had greater 1-, 2-, and 3-year survival rates (57.38%, 39.34%, and 29.51%) than the control group (32.79%, 18.03%, and 8.20%), with statistically significant differences (all *P* < 0.05).

**Conclusion:**

Microwave ablation in combination with an anti-PD-1 monoclonal antibody could effectively improve the level of T cell subsets and serum tumor markers in NSCLC patients, resulting in a long-term prognosis of patients with good therapeutic effect and safety.

## 1. Introduction

Among malignant tumor diseases, lung cancer is highly prevalent in China. With the elevated aggravation of air pollution, the prevalence of lung cancer also increases globally. Non-small-cell lung cancer (NSCLC) is responsible for approximately 85% of cases of lung cancer, according to statistics [1, 2]. Most of the patients had been in the advanced stage when diagnosed and had lost the chance of treatment via surgery. Systemic chemotherapy was mostly used, but its effect in improving the survival time of the patients is not satisfying. According to the relevant studies, programmed death-1 (PD-1) can be used as an immune checkpoint to inhibit T cell immune function by inhibiting the dephosphorylation of tyrosine phosphatase SHP-2 in the downstream signaling pathway of T cell antigen receptor. When T cells are repeatedly stimulated by the tumor microenvironment and chronic infection antigen, PD-1 expression level can be further promoted and T cell differentiation can be induced to enter the depletion state [3, 4]. Immunotherapy targeting immune checkpoint PD-1 and programmed death ligand-1 (PD-L1) inhibitors is a new treatment scheme for advanced lung cancer. PD-1 inhibitors such as pembrolizumab and nivolumab have achieved good clinical therapeutic effects [5, 6]. Immunotherapy is relatively safe compared with chemotherapy, but it may cause immune-related adverse reactions. In latest years, the clinical treatment of NSCLC has seen a significant increase in the use of percutaneous microwave curing therapy (PMCT). It has the benefits of good efficacy, high safety, and low trauma. Microwave heating can promote the coagulation and necrosis of tumor tissue, increase the permeability of cell membrane and nuclear membrane, and lead to the exposure of denatured and degraded single-stranded DNA complex, which is conducive to targeted treatment. Compared with traditional radiofrequency ablation, microwave ablation also has the advantage of ablating a large number of necrotic tissues in a short procedure time, which can better treat perivascular tissues and enlarge the ablation area [7]. This research sought to determine the impact of anti-PD-1 monoclonal antibody in combination with microwave ablation on the level of T cell subsets and the long-term prognosis of NSCLC.

## 2. Material and Methods

### 2.1. General Data

A total of 122 NSCLC patients who received treatment at our hospital between May 2015 and June 2019 were selected and assigned to the observation group and the control group by employing the random number table technique. Each group comprised 61 patients (*n* = 61). The observation group consisted of 22 females and 39 males. The average age was 59.67 ± 7.61 years, with ages ranging from 32 to 82. According to the histopathological classification of the patients, there were 37and 24 cases of adenocarcinoma and squamous cell carcinoma, respectively. TNM staging revealed that 13 patients were in stage I, 9 were in stage II, 16 were in stage III, and 23 were in stage IV. In 39 patients, the tumor was found in the right lung, while in 22 patients, it was found in the left lung. There were 26 patients who had tumors larger than 3 cm and 35 patients whose tumors were smaller than or equal to 3 cm. There were 25 females and 36 males in the control group. The mean age was 59.44 ± 7.63, with ages ranging from 30 to 83. As per the histopathological classification of the patients, there were 39 and 22 cases of adenocarcinoma and squamous cell carcinoma, respectively. There were 36 patients with tumors in the right lung and 25 patients with tumors present in the left lung, with 16 patients having stage I, 12 patients having stage II, 13 patients having stage III, and 20 patients had stage IV as per TNM staging. There were 31 patients suffering from tumors larger than 3 cm and 30 patients with tumors smaller than or equal to 3 cm. The two groups' general data were comparable (*P* > 0.05). The Hospital Ethics Committee provided their approval for this research.

### 2.2. Inclusion Criteria

(1) The diagnosis of NSCLC patients was made by clinicopathological examination [8]; (2) the Karnofsky Performance Status (KPS) score was >60; (3) life expectancy was >6 months; (4) all patients signed their informed consent and volunteered to take part in the study.

### 2.3. Exclusion Criteria

(1) Patients suffering from cardiopulmonary dysfunction; (2) patients having other malignant tumor diseases; (3) patients with severe hepatic and renal insufficiency; (4) patients with serious cardiovascular and cerebrovascular diseases; (5) patients with a history of pulmonary fibrosis or interstitial disease; (6) patients having a history of infusion reaction after antibody treatment; (7) patients with uncorrected thrombocytopenia or coagulopathy.

### 2.4. Methods

The control group received an anti-PD-1 monoclonal antibody and the observation group received microwave ablation in combination with an anti-PD-1 monoclonal antibody.

#### 2.4.1. Microwave Ablation

The patient was fasted for 6 h before surgery. Half an hour before surgery, the patient was given 0.5 mg atropine sulfate, 10 mg diazepam intramuscular injection, and 30 mg codeine tablet oral treatment. Ten minutes before surgery, the patient was given a 10 mg bucinperazine intramuscular injection. The puncture point, direction, and depth of the needle were determined according to the tumor site revealed by the recent chest CT, and the puncture point was marked on the surface of the chest wall. At the puncture site, local anesthesia was administered using 5–15 mL of 1% lidocaine. The patient was told to hold his breath, and the microwave ablation antenna was inserted at the predetermined site and heated for 3-5 min at the power of 60-75 W. When the tumor diameter was smaller than or equal to 3 cm, one-point ablation was given; and when the maximum tumor diameter was greater than 3 cm, single-needle multipoint ablation or multineedle ablation was given according to the tumor shape. For tumor > 3 cm, the ablation range was 0.5-1.0 cm beyond the tumor edge, and it was appropriate when there was a ~0.5 cm wide ground glass reaction zone around the tumor on the lung window. During and 12 h after surgery, symptomatic treatments, including ECG monitoring, oxygen inhalation, blood oxygen saturation detection, intermittent listening to double-lung breath sounds, infection prevention, and hemostasis, were given to the patient. On day 1 postoperatively, a chest X-ray examination was performed to observe whether the patient had pneumothorax, liquid pneumothorax, and other complications.

#### 2.4.2. Anti-PD-1 Monoclonal Antibody Therapy

The patient was treated by intravenous infusion of nivolumab injection (Bristol-Myers Squibb holdings Pharma, Ltd. Liability Company, USA, Registration Certificate No.: S20180014) at a dose of 3 mg/kg for 60 min. The treatment lasted for 6 cycles, with a drip every 14 days.

### 2.5. Observational Indices

(1) Clinical efficacy: the curative effects of the two groups were evaluated according to the response evaluation criteria in solid tumors RECISTI.1, which included complete remission (CR), partial remission (PR), stable disease (SD), and progressed disease (PD). CR: the patient's lesion disappeared entirely, and the maintenance period lasted more than 4 weeks; PR: more than 30% of the lesion's diameter was shortened, and the maintenance period lasted 4 weeks; SD: the curative effect failed to meet PR and PD standards; PD: the tumor's total length and diameter grew by more than or equal to 20%, or new lesions developed. Response rate (RR) = (CR + PR)/total number of cases × 100%. Total effective rate = significant effective + effective. (2) Levels of T cell subsets: five milliliters of fasting venous blood was drawn from each patient in the two groups before and after treatment. The blood was subjected to centrifugation for 15 minutes at 3000 rpm to separate the serum. The levels of T cell subsets (CD3+, CD4+, and CD8+) were measured via flow cytometry according to the operation instructions. (3) Serum tumor markers: the levels of squamous cell carcinoma antigen (SCCA), cytokeratin Ig fragment (CYFRA21-1), and carcinoembryonic antigen (CEA) in serum were determined by electrochemiluminescence immunoassay. (4) Appropriate amount of cancer cells was extracted by percutaneous puncture, and RNA was extracted by extraction kit. Extraction and reverse transcription were performed with reverse transcription kits. The nuclear factor kappa B (NF-*κ*B), protease C (PKC), and mitogen-activated protein kinases (MAPK) genes were amplified by PCR kit. The kits were obtained from SBS Genetech Co., Ltd. (Beijing, China). Prior to and following the treatment, a comparison was drawn between the two groups mRNA expression levels of NF-*κ*B, PKC, and MAPK. (5) Long-term prognosis: telephone and outpatient services were employed for carrying out follow-up. In the first year, follow-ups were conducted once per month; in the second and third years, they were conducted once every three months and once every six months, respectively. The two groups' survival times were noted, and the survival of both groups was analyzed via the Kaplan-Meier method. (6) Occurrence of adverse reactions: the WHO criteria were used for evaluating the adverse reactions. Adverse reactions were classified into levels 0 to 4. The incidence of digestive tract reaction, liver and kidney function impairment, bone marrow transplantation, hematotoxicity, and peripheral neurotoxicity were compared between both groups

### 2.6. Statistical Analysis

All the data of this survey were entered into Excel without communication between two people and processed with the statistical software SPSS24.0. Mean ± SD ($\bar{x}\pm \text{s}$) represented the measurement data. When the measurement data conformed to the normal distribution and the variance was homogeneous, a *t*-test was adopted. The counting data were described by cases and %. Fisher's exact probability method and the *χ*^2^ test were both utilized to compare the disordered classification data, and both tests were two-sided. *P* < 0.05 demonstrated statistical significance.

## 3. Results

### 3.1. Clinical Efficacy Comparison between the Two Groups

The observation group's RR was 80.33%, and the control group's RR was 62.30%, with statistically significant differences between the two groups (*P* < 0.05, Table 1).

### 3.2. Comparison of T Lymphocyte Subsets between the Two Groups

Prior to treatment, no considerable differences were observed between the two groups in regard to their CD3+, CD4+, or CD8+ levels (all *P* > 0.05). Upon treatment, the CD3+ and CD4+ levels increased and CD8+ levels reduced in both groups. The observation group's each index had an increased degree of improvement as compared to the control group, with statistically significant differences (*P* < 0.05, Table 2).

### 3.3. Comparative Analysis between the Two Groups' Serum Tumor Markers

Prior to treatment, no considerable differences were observed between the two groups in regard to their serum levels of CYFRA21-1, SCCA, or CEA (all *P* > 0.05). Following treatment, both groups' serum levels of SCCA, CYFRA21-1, and CEA decreased, and the observation group's indices were lesser as compared to the control group, with significant differences (*P* < 0.05, Table 3).

### 3.4. Comparison of Expression Levels of NF-*κ*B, PKC, and MAPK mRNA between the Two Groups

There were no considerable differences between the two groups mRNA expression levels of NF-*κ*B, PKC, and MAPK, prior to treatment (all *P* > 0.05). Following the treatment, the expression levels of NF-*κ*B mRNA, PKC mRNA, and MAPK mRNA of both groups were reduced, and the observation group's indices were lesser than those of the control group, with significant differences (all *P* < 0.05, Table 4).

### 3.5. Comparison of the Two Groups' Survival Time

The observation groups' 1-, 2-, and 3-year survival rates (57.38%, 39.34%, and 29.51%) were greater than the control group (32.79%, 18.03%, and 8.20%), with statistically significant differences (all *P* < 0.05; Table 5 and Figures 1–3).

### 3.6. Comparison Analysis of Adverse Reactions between the Two Groups

No considerable differences were observed in the occurrence of gastrointestinal reaction, liver and kidney function impairment, bone marrow suppression, hematotoxicity, and peripheral neurotoxicity between both the groups (all *P* > 0.05, Table 6).

## 4. Discussion

Percutaneous microwave ablation is a relatively safe minimally invasive treatment. The only common contraindications are uncorrectable thrombocytopenia and coagulation disorders, and the surgery can even be carried out in the clinic. Patients with pulmonary dysfunction may experience a temporary exacerbation of respiratory symptoms prior to treatment and require oxygen therapy for a period of time [9]. Microwave ablation is a local treatment. For patients having peripheral lung cancer with tumor diameter < 3 cm, a single-needle ablation can completely inactivate the tumors. However, for tumors with a diameter > 5 cm, many residues remain after treatment, which may lead to tumor recurrence [10]. Multipoint, multidirectional, and multilevel microwave ablation should be applied to tumors with a diameter ≥ 3 cm, and the inactivation range should be extended to 0.5-1.0 cm beyond the tumor edge as far as possible. However, distant metastasis or lymph node metastasis usually exists in advanced lung cancer, so microwave ablation alone is not suitable for the treatment of this kind of tumor. PD-1 is an important immune checkpoint and is a protective molecule of the body's immune system. By interacting with PD-L1, PD-1 can inhibit the inflammatory damage caused by T cell overactivation and effectively maintain the body's peripheral tolerance. Utilizing this characteristic, tumor cells overexpress immune checkpoint molecules to inhibit human immune system response, escape immune surveillance, and promote tumor cell growth [11, 12]. The immunosuppressive tumor microenvironment can activate the PD-1/PD-L1 signaling pathway, and blocking the PD-1/PD-L1 signaling pathway reverses the tumor immune microenvironment and increases the body's immune system's capability of killing the cancerous cells. The anti-PD-1 monoclonal antibody can effectively block the PD-1/PD-L1 signaling pathway. In the present study, the observation groups' patients received microwave ablation in combination with the anti-PD-1 monoclonal antibody, so that the efficacy of microwave ablation can be enhanced and the effect of immunotargeted therapy can be fully played to. In this study, RR (80.33%) in the observation group was substantially elevated than the RR of the control group (62.30%) following the treatment, and the improved levels of CD3+, CD4+, and CD8+ in the observation group were greater than the control group after treatment, implying that microwave ablation in combination with anti-PD-1 monoclonal antibody was superior to the lone use of anti-PD-1 monoclonal antibody for treating the NSCLC and can enhance the patients' cellular immunity in a more effective manner. CD3+ T lymphocytes can play an immune role in clearing tumor cells. CD4+ T lymphocytes, as auxiliary T cells, can not only play a direct killing role on tumor cells but also have immune memory function, playing a secondary immune role. CD8+ T lymphocytes are cytotoxic T lymphocytes, which can negatively regulate tumor immune response and can be used to evaluate the patient's autoimmune function [13, 14]. In the process of the development of NSCLC, apoptosis of tumor-specific T cells and PD-1-dependent and PD-1-independent mechanisms of mediation are closely related. PD-1-dependent mechanism can promote the immune escape of tumor cells in NSCLC patients. Peripheral blood T lymphocytes in NSCLC patients may show abnormal expression levels, including decreased CD3+ and CD4+ cells and increased CD8+ cells. Anti-PD-1 monoclonal antibody therapy can effectively improve the level of T lymphocytes in peripheral blood, relieve tumor load, and restore abnormal lymphocyte subsets [15]. Microwave ablation promoted tumor tissue necrosis and enhanced the effect of immunotherapy by improving the permeability of cell membrane and nuclear membrane. Therefore, the improvement effect of the T lymphocyte subgroup level in the observation group was better. Earlier research shows that microwave ablation can promote the patient's immune response to malignant tumors [16]. Our study's findings are in accordance with those of the earlier research.

Serum tumor markers refer to substances produced, secreted, or released by tumor cells into body fluid, blood, cells, or tissues that can reflect the presence and growth of the tumor. The expression level of serum tumor markers in normal or benign tissues is extremely low, and its level is highly associated with the incidence and progression of malignant tumors. Thus, it can reflect the case classification of tumor tissues and be used for disease analysis. As a soluble glycoprotein antigen, CEA is widely present in embryonic tumor and adenocarcinoma tissues, and its positive rate in lung adenocarcinoma is significantly higher than that in squamous cell carcinoma [17]. CYFRA21-1, the soluble fragment of cytokeratin Ig, is widely present in the cytoplasm of epithelial tumors such as esophageal cancer and lung cancer. It is a new tumor marker and can be used for the early diagnosis and prognosis of NSCLC [18]. Squamous cell carcinoma patients' serum contains significant amounts of SCCA [19]. The current research demonstrated that after treatment, serum levels of SCCA, CYFRA21-1, and CEA significantly decreased in the observation group in comparison to the control group, suggesting that anti-PD-1 monoclonal antibody and microwave ablation together could more effectively regulate the level of tumor markers. This may be because of the fact that the thermal effect of microwave ablation promotes irreversible necrosis of tumor tissue, destroys tumor cells in large quantities, and reduces the tumor load of the body. The combined therapy had an obvious tumor reduction effect, and the observation groups' level of serum tumor marker was more significantly reduced.

Previous research demonstrated that the PKC, MAPK, and NF-KB pathways are highly associated with the formation of VEGF. A series of cascade reactions among the three pathways can promote the synthesis and secretion of VEGF and promote tumor angiogenesis [20]. According to the current research, the NF-KB mRNA, PKC mRNA, and MAPK mRNA expression levels in the observation group were substantially enhanced as compared to the control group following the treatment, suggesting that microwave ablation in combination with anti-PD-1 monoclonal antibody may play a therapeutic effect by affecting PKC, MAPK, and NF-KB pathways, but there is no relevant clinical study at present. There, more research must be conducted to determine its precise mode of action. In this study, the observation group's 1-, 2-, and 3-year follow-up survival rates (32.79%, 18.03%, and 8.20%) were greater as compared to the control group (57.38%, 39.34%, and 29.51%), suggesting that combination therapy can more effectively enhance the patients' long-term prognosis.

In the current research, there were no considerable differences in the incidences of digestive tract reaction, liver and kidney function impairment, bone marrow suppression, hematotoxicity, and peripheral neurotoxicity between both groups. Although an additional treatment method was added to the observation group, adverse reactions were not aggravated, indicating that microwave ablation was safe.

In conclusion, percutaneous microwave ablation combined with an anti-PD-1 monoclonal antibody was effective in the treatment of NSCLC. This combined therapy could effectively improve the level of T lymphocyte subsets and long-term prognosis with good safety and clinical value.

## Figures and Tables

**Figure 1:** Survival curve of 1-year follow-up.

**Figure 2:** Survival curve of 2-year follow-up.

**Figure 3:** Survival curve of 3-year follow-up.

**Table 1:** Clinical efficacy comparison between the two groups (cases, %).

Group	CR	PR	SD	PD	RR
Observation group (*n* = 61)	29 (47.54)	20 (32.79)	8 (13.11)	4 (6.56)	49 (80.33)
Control group (*n* = 61)	20 (32.79)	18 (29.51)	14 (22.95)	9 (14.75)	38 (62.30)

*χ* ^2^					4.848
*P*					0.028

Note: CR: complete remission; PR: partial remission; SD: stable disease; PD: progressed disease; RR: response rate.

**Table 2:** Comparison of the two groups' T lymphocyte subsets ($\overset{¯}{x}\pm s$, %).

Group	CD3+		CD4+		CD8+	
	Before treatment	After treatment	Before treatment	After treatment	Before treatment	After treatment
Observation group (*n* = 61)	55.86 ± 5.70	67.41 ± 6.74^a^	36.73 ± 3.11	42.34 ± 3.45^a^	29.88 ± 2.49	20.74 ± 1.87^a^
Control group (*n* = 61)	55.18 ± 4.33	64.47 ± 6.08^a^	36.45 ± 3.07	40.16 ± 2.92^a^	29.44 ± 2.47	23.60 ± 2.16^a^

*t*	0.741	2.535	0.502	3.777	0.989	7.814
*P*	0.460	0.013	0.617	<0.001	0.325	<0.001

Note: compared to the same group's pretreatment data, ^a^*P* < 0.05.

**Table 3:** Comparison of serum tumor markers between the two groups ($\overset{¯}{x}\pm s$).

Group	SCCA (ng/mL)		CYFRA21-1 (μg/L)		CEA (μg/L)	
	Before treatment	After treatment	Before treatment	After treatment	Before treatment	After treatment
Observation group (*n* = 61)	9.50 ± 0.94	3.57 ± 0.56^a^	26.55 ± 2.74	12.80 ± 2.37^a^	66.07 ± 5.46	42.50 ± 4.38^a^
Control group (*n* = 61)	9.66 ± 0.99	5.73 ± 0.64^a^	25.91 ± 2.47	16.33 ± 3.08^a^	67.98 ± 5.40	46.35 ± 4.52^a^

*t*	0.911	19.867	1.348	7.036	1.939	4.765
*P*	0.364	<0.001	0.180	<0.001	0.055	<0.001

Note: compared to the same group's pretreatment data, ^a^*P* < 0.05.

**Table 4:** Comparison of expression levels of NF-*κ*B, PKC, and MAPK mRNA between the two groups ($\overset{¯}{x}\pm s$).

Group	NF-*κ*B mRNA		PKC mRNA		MAPK mRNA	
	Before treatment	After treatment	Before treatment	After treatment	Before treatment	After treatment
Observation group (*n* = 61)	0.91 ± 0.19	0.24 ± 0.12^a^	0.90 ± 0.14	0.24 ± 0.11^a^	0.93 ± 0.14	0.21 ± 0.11^a^
Control group (*n* = 61)	0.90 ± 0.11	0.53 ± 0.12^a^	0.91 ± 0.12	0.45 ± 0.15^a^	0.92 ± 0.14	0.48 ± 0.14^a^

*t*	0.446	13.325	0.337	8.469	0.322	11.795
*P*	0.656	<0.001	0.737	<0.001	0.748	<0.001

Note: compared to the same group's pretreatment data, ^a^*P* < 0.05.

**Table 5:** Comparison of the two groups' survival time (cases, %).

Group	Follow-up for 1 year		Follow-up for 2 years		Follow-up for 3 years	
	Survival	Death	Survival	Death	Survival	Death
Observation group (*n* = 61)	35 (57.38)	26 (42.62)	24 (39.34)	37 (60.66)	18 (29.51)	43 (70.49)
Control group (*n* = 61)	20 (32.79)	41 (67.21)	11 (18.03)	50 (81.97)	5 (8.20)	56 (91.80)

Log-rank *χ*^2^	7.980		9.039		11.210	
*P*	0.005		0.003		0.001	

**Table 6:** Comparison analysis of adverse reactions between the two groups (cases, %).

Group	Observation group (*n* = 61)			Control group (*n* = 61)			*χ* ^2^	*P*/Fisher's exact probability value
	I/II grade	III grade	Total incidence	I/II grade	III grade	Total incidence		
Gastrointestinal reaction	14 (22.95)	1 (1.64)	15 (24.59)	14 (22.95)	2 (3.28)	16 (26.23)	0.043	0.835
Liver and kidney function impairment	1 (1.64)	1 (1.64)	2 (3.28)	2 (3.28)	1 (1.64)	3 (4.92)	—	1.000
Bone marrow suppression	14 (22.95)	2 (3.28)	16 (26.23)	13 (21.31)	1 (1.64)	14 (22.95)	0.177	0.674
Hematotoxicity	7 (11.48)	1 (1.64)	8 (13.11)	4 (6.56)	0 (0.00)	4 (6.56)	1.479	0.224
Peripheral neurotoxicity	4 (6.56)	1 (1.64)	5 (8.20)	5 (8.20)	1 (1.64)	6 (9.84)	0.100	0.752

## Data Availability

The labeled dataset used to support the findings of this study is available from the corresponding author upon request.
